# Numerical Analysis of Nasal Flow Characteristics with Microparticles

**DOI:** 10.1155/2022/8706978

**Published:** 2022-08-22

**Authors:** Yi Liu, Wan Lin Sun

**Affiliations:** Faculty of Mechanical Engineering & Automation, Zhejiang Sci-Tech University, Hangzhou, China

## Abstract

This study was to investigate the airflow characteristics in nasal cavity under different conditions and analyze the effects of different respiratory intensity, particle diameter, and particle density on the deposition of particles carried by airflow in the nasal cavity, respectively. The three-dimensional geometric model of the nasal cavity was established based on typical medical images. The SST k-*ω* turbulence model in the computational fluid dynamics (CFD) was used to simulate the airflow in the nasal cavity, and the deposition of particles in the airflow was analyzed with the Lagrange discrete phase model. The results showed that the air in the nasal cavity flows in the left and right nasal passages through the perforation in front of the nasal septum and forms a vortex structure at the perforation site, and the particle deposition efficiencies (DE) under perforation nasal cavity are higher than that under normal nasal cavity. Different parameters had different effects on the particle DE. The results showed that the DE of particles with smaller size (≤2.5 *μ*m) is lower; the higher the respiration intensity, the greater the influence on the DE of the larger particle size; and the larger particle density (>1550 kg·m^−3^) has little effect on the DE of larger particle size (DP = 10 *μ*m). The results agree well with the corresponding research data.

## 1. Introduction

By the end of February 2022, there were more than 400 million confirmed COVID-19 cases and more than 5.9 million deaths worldwide, including more than 100,000 confirmed cases in China [1]. As a respiratory infectious disease, respiratory particle transmission and contact transmission are considered to be the main routes of transmission of COVID-19 [2]. Although measures such as high levels of protection for health-care workers (such as wearing N95 masks) and promotion of ventilation were targeted at airborne transmission routes, the importance of airborne transmission remains highly controversial. Meanwhile, human annual production activities release a large number of microparticles into the atmosphere [3, 4], its composition is complex, and microarticles in the air fuse with bacteria and viruses form biologically active particles. Atmospheric particles are light in weight and small in size, which are easily transmitted in the air and deposited in the human respiratory system through respiration, leading to chronic diseases [5, 6].

Nasal septum perforation is one of the common clinical diseases. With the development and maturity of nasal endoscopic surgery techniques, the incidence of iatrogenic nasal septal perforation gradually increased, accounting for 0.7–1.4% of patients undergoing nasal endoscopic surgery [7]. In recent years, due to the application of nasal spray hormone and nasal spray decongestant, the local microenvironment of the nasal septum has changed, and the cases of nasal septum perforation have gradually increased. Meanwhile, bioactive microparticles in the environment may aggravate the condition of patients with nasal septum perforation. After nasal septum perforation, mild cases have no clinical manifestations and the normal life of patients will not be affected, while severe cases will not only lead to nasal ventilation function decline but also cause different degrees of clinical symptoms, bringing trouble to the life of patients. In recent years, biological numerical simulation has a significant advantage in the study of nasal physiological function and pathogenesis and can intuitively show the effect of nasal structural changes on ventilation function. Therefore, it is of great scientific significance to study the deposition of microparticles in the human respiratory system through numerical simulation.

By simulating airflow in the nasal cavity of 22 healthy adults, Zhao et al. [8] found that there were significant differences in respiratory patterns and characteristics of healthy people. Therefore, this paper tends to study the upper respiratory tract in specific individual models. Researchers have carried out many studies on airflow and particles in the respiratory tract. Gabory et al. [9] used computational fluid dynamics to simulate repeated circular breathing in the whole nasal cavity, and the pressure gradient in the sinus cavity changed according to its connection position with the main passage. By establishing a three-dimensional numerical model of the normal human respiratory tract, Shen et al. [10] simulated the distribution of airflow and particles in the respiratory tract during the inspiratory process. Tsutomu et al. [11] used a numerical model to simulate the repair operation of nasal septum perforation. Xiong et al. [12] simulated the maxillary sinus open surgery. Lindemann et al. [13] studied the changes in nasal physiological environment before and after turbinectomy. Shen et al. [14] selected 9 normal people and 2 patients with nasal septum deviation (before and after surgery) as the research objects to establish a three-dimensional finite element model of the nasal cavity and obtained the airflow distribution, airflow temperature, and humidity in the nasal airway through numerical simulation and compared the results of numerical simulation between normal people and patients, as well as between patients before and after surgery. Jayaraju et al. [15] used Sension 16 CT scanner to carry out multislice CT imaging in 5 healthy men (who had never smoked) and Amira 4.0 software to perform 3d reconstruction of geometry. The deposition simulation of particles was simulated by CFD. Cheng et al. [16] used silicone materials to build a three-dimensional model of the upper respiratory tract based on the size of the volunteers' respiratory tract. Kim et al. [17] experimentally studied the deposition characteristics of aerosol particles with a G3-G5 respiratory tract model made of glass tubes. Yang-yang et al. [18] studied the airflow condition of the upper respiratory tract by combining physical model and numerical simulation based on 3D printing and CT 3D reconstruction. Grgic et al. [19] used CT scanning to collect data of the human respiratory tract and established a simplified three-dimensional geometric model, which is also called the ARLA (Aerosol Research Laboratory of Alberta) model. Xiu Guo et al. [20] established a computer numerical simulation model of the human upper respiratory tract and used computational fluid dynamics to simulate aerosol deposition. These studies mainly simulated the airflow, temperature, and humidity in a normal nasal cavity and the nasal surgery process under specific conditions.

In this paper, the CFD method was used to simulate the movement of airflow from the environment and the deposition of airflow particles in nasal septum during respiration. This study focuses on the changes of airflow state caused by nasal structure changes and the influence on the movement of particle deposition, so as to obtain the rule of particle deposition and provide a certain basis for nasal treatment.

## 2. Research Methods

### 2.1. Nasal Cavity Model

The nasal cavity model used in this paper is shown in Figure 1. A 3D image of the nasal cavity was established based on typical medical images, and the Geomagic Studio 3D modeling software was used to further improve the derived geometry, resulting in a realistic 3D model of the nasal cavity. In order to simplify the boundary conditions of CFD model, the inlet and outlet of nasal cavity were reconstructed and set as airflow velocity inlet and pressure outlet, respectively.

The nasal valve region has important physiological and pathological significance in nasal respiratory function, and clinical observation also found that there were many nasal septum perforations at the front of the nasal cavity, including the nasal foramen, the corresponding position at the front of the middle turbinate, which had the greatest impact on patients, and relatively few patients were located in the middle and back of the nasal cavity. Therefore, a circular perforation with a diameter of 10 mm was created in the anterior lower part of the septum to establish the nasal cavity model in the perforated state of the septum.

### 2.2. Numerical Simulation Method

Assuming that the nasal airflow was steady, incompressible, and isothermal, the flow continuity and momentum equation can be expressed as

(1) $$\begin{array}{c} \frac{\partial u_{i}}{\partial x_{i}}=0,\\ u_{j}\frac{\partial u_{i}}{\partial x_{j}}=-\frac{1}{\rho }\frac{\partial P}{\partial x_{i}}+\frac{\partial }{\partial x_{j}}\left(\left(\nu +\nu_{t}\right)\frac{\partial u_{i}}{\partial x_{j}}\right), \end{array}$$

where *u*_*i*_ (*i* = 1,2,3) represents the velocity of airflow in space, *P* is the pressure of airflow, *ρ* is the airflow density, *x*_*i*_ (*i* = 1,2,3) is the coordinate direction in space, *ν* is the kinematic viscosity of airflow, and *ν*_*t*_ is the kinematic turbulent viscosity of the fluid.

The SST k-*ω* turbulence model in ANSYS Fluent was adopted in this paper. The model can accurately predict the turbulent kinetic energy *k* of the boundary, thus reducing the difference between isotropic and anisotropic pulsation velocity assumptions and improving the calculation accuracy [21]. The governing equation of the SST k-*ω* model is as follows:

(2) $$\begin{array}{c} \frac{\partial \left(\rho k\right)}{\partial t}+\frac{\partial \left(\rho ku_{i}\right)}{\partial x_{i}}=\frac{\partial }{\partial x_{j}}\left(\Gamma_{k}\frac{\partial k}{\partial x_{j}}\right)+G_{k}-Y_{k}+S_{k},\\ \frac{\partial \left(\rho \omega \right)}{\partial t}+\frac{\partial \left(\rho \omega u_{i}\right)}{\partial x_{i}}=\frac{\partial }{\partial x_{j}}\left(\Gamma_{\omega }\frac{\partial \omega }{\partial x_{j}}\right)+G_{\omega }-Y_{\omega }+D_{\omega }+S_{\omega }, \end{array}$$

where *G*_*k*_ represents the turbulent kinetic energy, Γ_*k*_ and Γ_*ω*_ represent the effective diffusion term of *k* and *ω*, *Y*_*k*_ and *Y*_*ω*_ represent the divergence term of *k* and *ω*, *D*_*ω*_ represents the orthogonal diffusion term, and *S*_*k*_ and *S*_*ω*_ are the user-defined source terms.

Airflow velocity *u*_*i*_ comprises of two components:

(3) $$\begin{array}{c} u_{i}={\bar{u}}_{i}+u_{i}^{\prime }, \end{array}$$

where ${\bar{u}}_{i}$ is the average velocity over time, and *u*_*i*_′ is the fluctuating component representing the randomly directed eddy. For the isotropic region, the fluctuating component *u*_*i*_′ can be calculated by

(4) $$\begin{array}{c} u_{i}^{\prime }=\xi_{i}\sqrt{\frac{2}{3}k}, \end{array}$$

where *ξ*_*i*_ are the random numbers from standard normal distribution. However, the DNS results indicated that the fluid in the near-wall region is anisotropic and that the fluctuating velocity of the fluid can be modeled by applying damping functions in different directions, i.e.,

(5) $$\begin{array}{c} u_{i}^{\prime }=f_{i}\xi_{i}\sqrt{\frac{2}{3}k}, \end{array}$$

(6) $$\begin{array}{c} f_{u}=1+0.285\left(y^{+}+6\right)\text{exp}\left[-0.455{\left(y^{+}+6\right)}^{0.53}\right], \end{array}$$

(7) $$\begin{array}{c} f_{v}=1-\text{exp}\left(-0.02y^{+}\right), \end{array}$$

(8) $$\begin{array}{c} f_{w}=\sqrt{3-f_{u}^{2}-f_{v}^{2}}, \end{array}$$

where *f*_*u*_ is the function for stream-wise direction, *f*_*v*_ is normal to the closest wall, and *f*_*w*_ is vertical to *f*_*u*_ and *f*_*v*_. Equations (6) ∼ (8) were applied for areas where the *y*^+^ values were less than 80. *y*^+^ is a dimensionless wall distance defined as

(9) $$\begin{array}{c} y^{+}=\frac{y}{\nu }\sqrt{\frac{\tau_{w}}{\rho }}, \end{array}$$

where *y* is the distance to the nearest wall and *τ*_*w*_ is the wall shear stress.

Because of the small volume rate of particles in the airflow, the Lagrange discrete phase model can be used to calculate and track the movement and deposition of particles after the flow field converges. The particles in the air could be regarded as tiny solid spherical particles. The discrete random walk model was used to simulate the effect of turbulence on the particles' motion. The motion of microparticles followed Newton's laws of motion, taking into account only the Saffman lift, drag, and gravity received by the microparticles. The motion equation of a single microparticle can be expressed as

(10) $$\begin{array}{c} m_{p}\frac{\text{d}u_{p}}{\text{d}t}=F_{G}+F_{D}+F_{S}, \end{array}$$

where *m*_*p*_ is the mass of the micro-particle, **u**_*p*_ is the velocity of the particle, **F**_*G*_ is the gravity of the particle, **F**_*D*_ is the drag force on the particle, and **F**_*S*_ is the Saffman force generated by the difference of fluid velocity on both sides of the particle.

The deposition efficiencies (DE) of microparticles can be expressed by the following equation:

(11) $$\begin{array}{c} \text{DE}=\frac{N_{t}}{N_{a}}\times 100\;\%, \end{array}$$

where *N*_*t*_ is the number of deposited microparticles and the total number of microparticles released is *N*_*a*_.

### 2.3. Boundary Condition

The respiratory airflow flow of a normal human body is a sine function that changes over time. Based on the steady-state hypothesis, the maximum airflow velocity at different respiratory intensities was used to simulate. The airflow velocity was obtained by (12), and the specific values are shown in Table 1.

(12) $$\begin{array}{c} u\left(t\right)=\frac{\text{d}Q\left(t\right)}{A\text{d}t}, \end{array}$$

where *u*(*t*) is the airflow velocity, *Q* is the respiratory intensity, *t* is the time, and *A* is the area of the nostril inlet.

The airflow inlet was located at the nostril (Figure 1), and the boundary type was set as the velocity inlet. Both airflow and particles entered the model perpendicular to the inlet plane. The flow outlet boundary type was defined as a pressure outlet (relative pressure = 0), and the other surface boundary types were defined as walls that can capture particles. The coupling mode between particles and airflow was one-way coupling, and the influence of particles on the flow field and the interaction between particles were ignored.

In numerical calculation, the deposition efficiencies of microparticles in a nasal cavity under different conditions were studied by changing the values of microparticle diameter (the selected particle size values are all within the range of acceptable particle size) and particle density (Table 2); the density of the absorbable particles ranges from 600 kg·m^−3^ to 2300 kg·m^−3^ [22–24].

### 2.4. Grid Independence

The nasal cavity model was divided by ICEM CFD software. According to the nasal cavity structure, the geometric model was divided by tetrahedral unstructured mesh. Three mesh numbers (1.8 million, 3.2 million, and 6.7 million) were used to divide the nasal cavity geometric model. The statistical results of velocity at different points in the nasal cavity are shown in Figure 2(a), and the ratio of the left and right nasal meatus flow (>0.90) was within the range of experimental data of Yang-yang et al. [18] (0.90∼0.95), as shown in Figure 2(b). In the comprehensive consideration of computing speed, computing equipment, and economic conditions, 3.2 million tetrahedral unstructured meshes were selected for numerical simulation and analysis. The calculation results tended to be stable and could meet the requirements of calculation accuracy. Numerical simulation was carried out in Fluent 2020 R1.

## 3. Results and Discussion

### 3.1. Airflow Field

As shown in Figure 3, the movement track of airflow into the nasal cavity is shown in the form of a streamline. The airflow trajectories of normal breathing (A), speaking (B), and coughing (C) are shown. It can be observed that in the stable state of inspiratory, the main airflow channels are the middle nasal meatus and the posterior end of the superior nasal meatus. Air flows from the nostrils straight into the middle nasal tract, and the air flows in a parabolic pattern inside the nasal cavity. The airflow in nasal septum perforation is different from that in a healthy nasal cavity. After entering the nasal cavity, the airflow flows from the left nasal tract to the right nasal tract through the nasal septum perforation, and there are some vortex structures in the nasal septum perforation.

According to the results of the streamline in the left nasal cavity, the airflow into the nasal cavity is relatively concentrated. The airflow enters the nasal cavity from the nostril, rushes straight to the front of the middle nasal tract, and then disperses. This is conducive to the rapid and adequate intake of air into the nasal cavity to the functional areas, while purifying the air. At the same time, compared with the normal condition of the nasal cavity, there are some obvious vortex structures due to the perforation of the nasal septum, which indicated that the airflow had shear or rotational motion. The existence of a vortex structure causes the airflow and the nasal cavity in the original perforated mucous membrane contact to be more frequent so the nasal septum perforated disease is more likely to aggravate. Combined with the study of Zubair et al. [25], these vortex structures are generated because of the uneven distribution of local pressure in the nasal cavity during respiration (Figure 3(c)).

### 3.2. Particle Deposition

The effect of particle size on the DE of particles in the nasal cavity is studied. As shown in Figure 4, the deposition of particles in the nasal cavity is simulated under the conditions of *ρ*_*p*_  = 1550 kg·m^−3^ and *Q* = 30 L·min^−1^. The minimum particle size is 0.25 *μ*m, and the maximum particle size is 10 *μ*m (the selected particle size values are all within the range of acceptable particle size). It can be seen that the DE of microparticles increased with the increase of particle size in the two nasal conditions. When the particle size is larger than 2.5 *μ*m, the DE of microparticles increases rapidly. The DE of a particle in the perforated nasal septum is higher than that in the normal nasal septum.

Then, we investigated the effect of density on the deposition of particles in the nasal septum by changing the density of particles in the two states. In Figure 5(a), when dp = 2.5, 5, 10 *μ*m, five different density values are set between 950 and 2150 kg·m^−3^ to obtain the DE of microparticles in the nasal septum under different nasal conditions. It can be seen that the DE of particles with different particle sizes is different with the increase in density. Under the condition of dp = 2.5 *μ*m, the DE of particles in normal nasal septum slowly increases with the increase of density. At a density greater than 1550 kg·m^−3^, it can be seen that the particle DE of nasal septum perforation is lower than that of the previous density conditions. When dp = 5 *μ*m, the DE of particles in the nasal septum is lower than that of particles in the nasal septum when dp = 2.5 *μ*m. It can be seen from the figure that the DE of particles in the nasal septum increases significantly in the density range of 1250∼1850 kg·m^−3^. When dp = 10 *μ*m, the particle DE of nasal septum perforated at the density of 1550 kg·m^−3^ is significantly higher than that of normal septum perforated at the density of 1550 kg·m^−3^. At a density greater than 1550 kg·m^−3^, the DE of the nasal septum is similar in the two conditions.

Figure 5(b) shows the effect of respiratory intensity on the deposition efficiencies of particles in the nasal septum at *Q* = 30, 60, 90 L·min^−1^, *ρ*_*p*_  = 1550 kg·m^−3^. When the respiration intensity is 30 L·min^−1^, the DE of 2.5 *μ*m and 5 *μ*m particles had little difference under different conditions, and the DEs of different particle sizes in the nasal septum are all higher in the perforation state than in the normal state. At 60 L·min^−1^ and 90 L·min^−1^, the particle DE in the normal state is higher than that in the perforation state. At the same time, the particle DEs in different states increase with the increase of respiration intensity.

When the airflow flows through the airway structure with drastic geometrical changes or large curvature, the particles are easily captured by the nasal surface mucus under the action of inertia. From the perspective of the nasal cavity structure, the nasal threshold is the bottleneck of the nasal cavity structure. When the airflow passes the nasal threshold into the nasal cavity, it contracts and expands, creating an area of microparticle deposition at a higher level in the inherent nasal front-end, where the septum is prone to perforation. Airflow changes at the perforated nasal septum also resulted in increased particle deposition efficiency in this area. Vecellio et al. [26] found in their study that the first area with a high concentration of microparticle deposition in the nasal cavity was about 2 cm away from the anterior nostril, located in the position of the inherent nasal front-end.

The deposition efficiencies of microparticles in different conditions are affected by particle size, density, and respiratory intensity. The inertia force of micron particles is the main influencing factor during the movement of micron particles in the respiratory tract. Therefore, with the increase in particle size and density, the DE of microparticles in the two nasal conditions is different. By comparison, it can be found that for the small particle size, the change of particle density has little influence on the DE of the particles, while the change in the nasal cavity has a great effect on it. Compared with the larger particle size, the change of particle density has a more obvious effect on the DE of microparticles, and with the increase of respiratory intensity, the velocity of airflow in the nasal cavity also increases, and the inertia of particle movement also increases. Therefore, the stronger the respiratory intensity, the higher the DE of particles will be. There is more variation in air velocity in the nasal cavity due to a perforated septum. As a result, particles in the airflow are more likely to come into contact with the nasal mucosa, further increasing the DE of particles in the nasal cavity. But, in the case of strong respiratory intensity, the particle DE of the nasal septum under perforation is lower than that under normal condition. Combined with Figure 4, it can be seen that the particle DE of other parts of the nasal cavity under perforation increased.

## 4. Conclusion

The airflow characteristics of the perforated nasal septum and normal nasal cavity were simulated under different respiratory intensities. The deposition efficiencies of particulate matter in the nasal cavity with the perforated septum and the normal nasal cavity were simulated under different particle size and particle density. The simulation results showed that the airflow in the nasal passages will flow in the left and right nasal passages through the septum perforation. The airflow velocity in the perforation was complex and variable. The results fit well with related experiments.

On the one hand, with the increase in particle size, the DE of particulate matter in the perforated nasal cavity was significantly higher than that in the normal nasal cavity, which indicates that the local nasal cavity condition in patients with a septum perforation is poorer. It can cause undesirable clinical symptoms to a certain degree, for instance, frequent headache, insomnia, dry nose, and repeated bleeding. On the other hand, with the increase in density, the DE of different particle sizes in the nasal septum varied. In the case of strong respiratory intensity, the DE of the nasal septum in the normal state was higher than that in the perforation state. This study compared the particle DE in the same part of the nasal cavity under different conditions, which is helpful for the prevention of nasal diseases and drug development of nasal administration therapy.

## Figures and Tables

**Figure 1:** Nasal cavity model and nasal septum perforation location diagram.

**Figure 2:** Numerical simulation and grid independence verification. (a) Airflow velocity at different points under different grid numbers. (b) Fluid flow and ratio of the left and right nasal meatus.

**Figure 3:** (a) Respiratory streamline diagram of normal nasal cavity. (b) Respiratory streamline diagram of perforated septum. (c) Pressure distribution at perforated septum.

**Figure 4:** The variation of particle DE with particle size.

**Figure 5:** Variation of particle DE in nasal septum under different conditions. (a) The variation of particle DE with particle density. (b) The variation of particle DE with respiratory intensity.

**Table 1:** Airflow velocity corresponding to different respiratory intensity.

Physiological state	Q/l·min^−1^	U/m·s^−1^
Normal breathing	30	3.44sin(*t∗π*/2)
Speech	60	6.88sin(*t∗π*/2)
Cough	90	10.32sin(*t∗π*/2)

**Table 2:** Values of particle size and particle density.

Parameter	Value
Particle diameter, dp/*μ*m	0.25, 0.5, 1.0, 2.5, 5.0, 7.5, 10.0
Particle density, *ρ*_*p*_ /kg·m^−3^	950, 1250, 1550, 1850, 2150

## Data Availability

Data sharing is not applicable to this article as no datasets were generated or analyzed during the current study.
